The article "Athlete Health Status Assessment Based on Edge Computing Model and Large-Scale Multimedia Health Data Analysis" was retracted in 2023. Reasons: signs of a paper mill; suspected computer-generated content; unreliable results or conclusions; concerns about the data.

# Athlete Health Status Assessment Based on Edge Computing Model and Large-Scale Multimedia Health Data Analysis

**DOI:** 10.1155/2022/1079663

**Published:** 2022-06-11

**Authors:** Xiaoyun Zhang

**Affiliations:** College of Vocal Language and Art, Sichuan University of Media and Communications, Chengdu, Sichuan 610000, China

## Abstract

This study explores the athlete's health status evaluation system based on an edge computing model and large-scale multimedia health data analysis in order to improve the assessment effect of athletes' current health state. In addition to that, this research builds a wireless signal propagation model in edge areas using bicubic polynomial interpolation, improves the accuracy of DEM data by using bicubic polynomial interpolation, and digitally represents the sports field by utilizing DEM data. In addition to that, the model and DEM data are utilized in this paper to realize the site selection process for base station networking. The experimental analysis demonstrates that the athletes' health status evaluation system suggested in this research, which is based on the edge computing model and the large-scale multimedia health data analysis, has a good effect on the assessment of athletes' health.

## 1. Introduction

The main purpose of establishing athlete health risk early warning and athlete health intervention management software is to provide an acquisition tool suitable for assisting self-body athlete health management and athlete health intervention guidance programs. This system uses the fully automatic whole body athlete health scanning system to examine the human body and obtain the physiological function parameters of the human body. Moreover, it combines the knowledge of basic medicine, clinical medicine, preventive medicine, and traditional Chinese medicine to establish a health risk assessment and early warning method for the eight major systems of the human body (respiratory system, digestive system, immune system, genitourinary system, exercise system, circulatory system, endocrine system, nervous system) and realizes early warning of the health risks of the eight major systems of athletes. In addition, a database of complete athlete health intervention measures for athletes' health problems in the eight major systems and major organs of the human body will be produced based on effective domestic and foreign measures. A computer data module was created from the first two study results, and a questionnaire survey module, an auxiliary inspection module, and a personal information input module were added. Athlete health risk warning and intervention management software can be developed using modern computer technologies at the same time. The software can realize early warning of athletes' health risks in various systems of the human body and query comprehensive athlete health intervention measures for athletes' health risk warning results. In addition, the computer assists doctors to formulate athletes' health intervention plans and follow-up visit plans, automatically generate user's athlete health risk warning reports and electronic athletes' health records, and use modern network technology to realize remote tracking of athletes' health interventions and other functions. This truly enables early warning and early intervention of health risks for athletes to prevent disease from occurring.

The article "Athlete Health Status Assessment Based on Edge Computing Model and Large-Scale Multimedia Health Data Analysis" was retracted in 2023. Reasons: signs of a paper mill; suspected computer-generated content; unreliable results or conclusions; concerns about the data.

A perfect athlete health intervention program also targets various aspects including living habits, diet, thinking, character, values, interpersonal relationships, family relationships, and home environment. The appropriate intervention measures are selected according to the actual conditions of the examinee, and finally an intervention plan that conforms to the examinee is formed.

Edge computing and large-scale multimedia health data analysis are used in this work to study the athlete's health status assessment system and improve the accuracy of subsequent health assessments.

## 2. Related Work

The remote monitoring system for pose and human health parameters is a wireless medical monitoring network. As a special medical monitoring, the function and performance of the monitoring system need to meet the needs of athletes and medical staff at the same time. The system mainly includes three aspects: data acquisition, wireless transmission, and long-distance communication between the master node and the personal monitoring terminal [1]. Data collection should take into account the convenience, nondisturbance, and certain emergency of collecting data. Simply put, the collected information should be easy to extract, can better reflect the physical health status of the collected object, and should not cause inconvenience to the life of the collected object [2]. In addition, it is necessary to make good and rapid emergency responses to some emergencies to ensure that the collected objects can receive the first-time healthcare and assistance. Wireless technology should comprehensively consider the following conditions: the length of communication distance, whether mobile communication can be realized, data transmission rate, suitable size, cost, preferably low transmission power, strong anti-interference ability, etc. [3]. Only when these conditions are well considered can the wireless medical monitoring network realize its function. The communication interface between the master node and the computer should be suitable for most computers, and the speed can meet the requirements [4]. In view of the fact that athletes and medical staff or guardians are generally not in the same place in daily life, the data is transmitted remotely, so that medical staff and guardians can understand the situation of the ward in real time, so that the ward can be given timely treatment when abnormal conditions occur [5].

The article "Athlete Health Status Assessment Based on Edge Computing Model and Large-Scale Multimedia Health Data Analysis" was retracted in 2023. Reasons: signs of a paper mill; suspected computer-generated content; unreliable results or conclusions; concerns about the data.

ZigBee health monitoring can provide safe, robust, high-performance, and fast wireless connection and operation for the user's physical condition and indoor and outdoor facilities and can use various devices around the world according to local conditions [6]. The cost-effective features of ZigBee in health monitoring have been recognized by the relevant industry and provide a safe, robust, high-performance wireless connection for the monitoring of athletes' activities and facilities, while providing freedom of wireless operation outdoors [7]. ZigBee health monitoring can utilize a wide variety of devices around the world and is particularly suitable for low-power LAN applications [8]. ZigBee health monitoring is available in a variety of cost-effective, industry-proven chip platforms that run on many of the world's largest semiconductor manufacturers. Healthcare services based on ZigBee technology enable the goal of safe and reliable monitoring and emergency treatment with an interoperable wireless device based on a global standard [9]. The service feeds back some effective physical health conditions of users, which can promote users to understand their own health conditions and actively improve them. It is suitable for families, community health centers, and hospitals. It can meet the various needs of different consumers and has a wide range of applicability [10].

The information acquisition module is mainly responsible for collecting mobile phone sensor information, including angular velocity information (responsible for the gyroscope), light intensity information (responsible for the light sensor), acceleration information (responsible for the accelerometer), and geomagnetic information (responsible for the geomagnetic sensor). This module provides data support for the operation of the upper-layer core subsystems [11]; the transmission module is mainly responsible for the data interaction between the client and the back-end server, and the exchanged information mainly includes user heat consumption ranking information, friend-related information, etc. [12]; the activity recognition subsystem is mainly used to reliably identify the user's basic activities and provide activity information for the quality of life assessment subsystem, including the type of activity and its duration [13]; the quality of life assessment subsystem integrates activity information as well as diet, weight, height, gender, and other information to judge whether the user's life is in a healthy state [14].

The article "Athlete Health Status Assessment Based on Edge Computing Model and Large-Scale Multimedia Health Data Analysis" was retracted in 2023. Reasons: signs of a paper mill; suspected computer-generated content; unreliable results or conclusions; concerns about the data.

The development of the system platform needs to follow certain design principles, but many factors need to be considered before the development of the system platform, including user needs, technical conditions, technical level, practicability, scientificity, etc. Some of these factors restrict each other, and some promote each other [15–17]. Therefore, in the design and construction process of the entire system, comprehensive consideration of many industry-leading technologies and popular trends, and based on the understanding and experience of software system construction, let the athlete health risk early warning and athlete health intervention management software systems be mature software. Based on the framework, it is implemented and developed in combination with specific needs [18]. Make the system have a high-stability and advanced core, ensure that the whole system has very good openness and integratability, support large load capacity, and at the same time have the forward-looking technology, which is in line with the popular development trend of the industry and can guarantee the project's implementation completion time, reducing the risk of project implementation [19]. Today's Internet software development is nothing more than the use of two architectures, BIS and C/S architecture, each with their own advantages. The C/S structure is a relatively traditional model. The client software and server software are deployed on the client and server, respectively, and the communication between the client and the server is handled through a network connection in the middle. The client of the software can help the system to complete the calculation process of most data, so the amount of data transmitted will be relatively small, and the network load will be relatively light. At the same time, because the client has already processed a part of the data, the amount that the server needs to process has also been reduced, and the load pressure of the server will not be reduced [20, 21].

## 3. Analysis and Design of Motion Evaluation Model Based on Edge Computing

In this paper, Digital Elevation Model (DEM) is used to quantitatively represent the pose [22, 23]. DEM data represents a finite sequence of three-dimensional column vectors in a certain region, and its functional expression is

(1) $$\begin{array}{c} v_{i}=\left(x_{i},y_{i},z_{i}\right);i=1,2,\ldots n. \end{array}$$

Among them, *v*_*i*_ represents the digital elevation vector, and *x*_*i*_, *y*_*i*_, *z*_*i*_ represent the abscissa, ordinate, and elevation value of the digital elevation data point, respectively.

The article "Athlete Health Status Assessment Based on Edge Computing Model and Large-Scale Multimedia Health Data Analysis" was retracted in 2023. Reasons: signs of a paper mill; suspected computer-generated content; unreliable results or conclusions; concerns about the data.

The representation models of DEM mainly include regular grid representation model, contour model representation, and irregular triangulation representation.

DEM data can be seen as connected by an infinite number of polynomial surfaces. When an *n*-th degree polynomial surface and its adjacent surfaces have continuous *n* − 1 derivative functions on the boundary, it is called a spline function. Based on the spline function, the bicubic polynomial (binary spline function interpolation method) can be used to improve the model resolution and accuracy. The expression for the bicubic polynomial is

(2) $$\begin{array}{c} z=\left[\begin{array}{cccc} 1 & x & x^{2} & x^{3} \end{array}\right]\left[\begin{array}{cccc} a_{00} & a_{01} & a_{02} & a_{03}\\ a_{10} & a_{11} & a_{12} & a_{13}\\ a_{20} & a_{21} & a_{22} & a_{23}\\ a_{30} & a_{31} & a_{32} & a_{33} \end{array}\right]\left[\begin{array}{c} 1\\ y\\ y^{2}\\ y^{3} \end{array}\right]=\bar{X}A{\bar{Y}}^{T}. \end{array}$$

Among them, *x*, *y*, and *z* are the abscissa, ordinate, and elevation values of the sampling points in the DEM data, respectively.

The partial derivative of *z* with respect to *x* is

(3) $$\begin{array}{c} z_{x}=\left[\begin{array}{cccc} 0 & 1 & 2x & 3x^{2} \end{array}\right]A{\left[\begin{array}{cccc} 1 & y & y^{2} & y^{3} \end{array}\right]}^{T}. \end{array}$$

The partial derivative of *z* with respect to *y* is

(4) $$\begin{array}{c} z_{y}=\left[\begin{array}{cccc} 1 & x & x^{2} & x^{3} \end{array}\right]A{\left[\begin{array}{cccc} 0 & 1 & 2y & 3y^{2} \end{array}\right]}^{T}. \end{array}$$

The second-order mixed partial derivative of *Z* with respect to *XY* is

(5) $$\begin{array}{c} z_{xy}=\left[\begin{array}{cccc} 0 & 1 & 2x & 3x^{2} \end{array}\right]A{\left[\begin{array}{cccc} 0 & 1 & 2y & 3y^{2} \end{array}\right]}^{T}. \end{array}$$

At the same time, there are the following relations in the unit grid:

(6) $$\begin{array}{c} \left\{\begin{array}{c} x_{i-1}=y_{i-1}=-1\\ x_{i}=x_{i}=0\\ x_{i+1}=y_{i+1}=1\\ x_{i+2}=y_{i+2}=2 \end{array}\right). \end{array}$$

Then, we can get

(7) $$\begin{array}{c} \bar{Z}=\left[\begin{array}{cccc} {\left(z\right)}_{i,j} & {\left(z_{y}\right)}_{i,j} & {\left(z\right)}_{i,j+1} & {\left(z_{y}\right)}_{i,j+1}\\ {\left(z_{x}\right)}_{i,j} & {\left(z_{xy}\right)}_{i,j} & {\left(z_{x}\right)}_{i,j+1} & {\left(z_{xy}\right)}_{i,j+1}\\ {\left(z\right)}_{i+1,j} & {\left(z_{y}\right)}_{i+1,j} & {\left(z\right)}_{i+1,j+1} & {\left(z_{y}\right)}_{i+1,j+1}\\ {\left(z_{x}\right)}_{i+1,j} & {\left(z_{xy}\right)}_{i+1,j} & {\left(z_{x}\right)}_{i+1,j+1} & {\left(z_{xy}\right)}_{i+1,j+1} \end{array}\right]\\ =\left[\begin{array}{cccc} 1 & 0 & 0 & 0\\ 0 & 1 & 0 & 0\\ -3 & -2 & 3 & -1\\ 2 & 1 & -2 & 1 \end{array}\right]A\left[\begin{array}{cccc} 1 & 0 & 0 & 0\\ 0 & 1 & 0 & 0\\ -3 & -2 & 3 & -1\\ 2 & 1 & -2 & 1 \end{array}\right]=\bar{X}A{\bar{Y}}^{T}. \end{array}$$

Among them, there is

(8) $$\begin{array}{c} {\bar{X}}^{-1}={\bar{Y}}^{-1}=\left[\begin{array}{cccc} 1 & 0 & 0 & 0\\ 0 & 1 & 0 & 0\\ -3 & -2 & 3 & -1\\ 2 & 1 & -2 & 1 \end{array}\right]. \end{array}$$

Then, there is $A={\bar{X}}^{-1}\bar{Z}{\bar{Y}}^{-T}$. Then, according to the calculation method of the derivative of *z*, there is

(9) $$\begin{array}{c} \left\{\begin{array}{c} {\left(z_{x}\right)}_{i,j}=\frac{\partial z_{i,j}}{\partial x}=\frac{1}{2}\left({\text{z}}_{i+1,j}-z_{i-1,j}\right),\\ {\left(z_{y}\right)}_{i,j}=\frac{\partial z_{i,j}}{\partial y}=\frac{1}{2}\left({\text{z}}_{i,j+1}-z_{i,j-1}\right),\\ {\left(z_{xy}\right)}_{i,j}=\frac{\partial^{2}z_{i,j}}{\partial x\partial y}=\frac{1}{4}\left({\text{z}}_{i+1,j+1}+{\text{z}}_{i-1,j-1}-z_{i-1,j+1}-z_{i+1,j-1}\right). \end{array}\right) \end{array}$$

It can be obtained that when the slopes and twists of *z* in the *x* and *y* directions at the grid points are equal, the boundary line has the same slopes along the *x* and *y* directions; that is, it is smooth. Finally, according to the value of the 16 grid points around the value point, the elevation value of the point to be measured can be obtained:

(10) $$\begin{array}{c} z=\sum_{i=0}^{3}\sum_{j=0}^{3-i}a_{ij}x_{i-1}y_{j-1}. \end{array}$$

Adopting the interpolation procedure results in a denser distribution of elevation points in a region of the same size. With a denser elevation point, the pose may be fitted with greater precision. The error calculation indicators such as mean error (MAE), mean square error (RMSE), and fit superiority (*R*^2^) are used to quantify the fitting error after interpolation in order to analyze the error between the DEM data and the original data after the interpolation calculation and the true posture. The calculation formula is as follows:

(11) $$\begin{array}{c} \text{MAE}=\frac{1}{n}\sum_{i=1}^{n}\left|{\hat{z}}_{i}-z_{i}\right|,\\ \text{RMSE}=\sqrt{\frac{1}{n}\sum_{i=1}^{n}{\left({\hat{z}}_{i}-z_{i}\right)}^{2}},\\ {\text{R}}^{2}=1-\frac{\sum_{i=1}^{n}{\left({\hat{z}}_{i}-z_{i}\right)}^{2}}{\sum_{i=1}^{n}{\left({\hat{z}}_{i}-\bar{z}\right)}^{2}}. \end{array}$$

Among them, ${\hat{z}}_{i}$ is the calculated elevation after the sampling point i's value, *z*_*i*_ is the real elevation of the sampling point *i*, and $\bar{z}$ is the average value of the actual elevation. *n* is the number of sampling points.

The article "Athlete Health Status Assessment Based on Edge Computing Model and Large-Scale Multimedia Health Data Analysis" was retracted in 2023. Reasons: signs of a paper mill; suspected computer-generated content; unreliable results or conclusions; concerns about the data.

The value of wireless signal transmission strength is dBm, and its calculation formula is

(12) $$\begin{array}{c} dBm=10\;\log\left(\frac{pout}{1mW}\right). \end{array}$$

Among them, Pout is the power value in mW. In an unobstructed environment, the propagation of wireless signals can be regarded as propagation in free space. The so-called free-space propagation refers to the propagation of radio waves when there is an infinite vacuum around the antenna, which is an ideal propagation condition. When a radio wave propagates in free space, its energy is neither absorbed by obstacles nor reflected or scattered. The communication distance is related to transmit power, receiver sensitivity, and operating frequency, and the propagation loss *L*_free_ in free space is given by formula (13).

(13) $$\begin{array}{c} L_{\text{free}}=32.4+20\;\log_{10}\left(f\right)+20\;\log_{10}\left(d\right). \end{array}$$

Among them, *d* represents the distance from the transmitter of the wireless signal to the receiver, and the unit is km. *f* is the radio frequency in MHz.

However, when the wireless signal is propagated in line-of-sight conditions near the ground surface, the formula for free-space signal propagation will be greatly deviated due to the influence of the ground reflection. Therefore, ground reflections need to be taken into account for path loss. According to Okumura's empirical model, the earth plane path loss model is obtained as

(14) $$\begin{array}{c} L_{PE}\left(dB\right)=40\;\log_{10}\left(d\right)-20\;\log_{10}\left(h_{T}\right)-20\;\log\left(h_{R}\right). \end{array}$$

Among them, *d* is the distance between the isotropic signal transmitting device and the receiving device. *h*_*T*_ and *h*_*R*_ are the heights of the wireless signal transmitting device and the wireless signal receiving device from the ground, respectively. In this formula, it needs to require *d* to be much larger than *h*_*T*_ and *h*_*R*_. Formulas (15) and (16) and the antenna gain loss in the Okumura model are combined; we get the wireless signal propagation loss model in the open pose:

(15) $$\begin{array}{c} L_{M}=L_{\text{free}}+A_{m}\left(f,d\right)-H_{T}\left(h_{T},d\right)-H_{R}\left(h_{R},f\right). \end{array}$$

Among them, *L*_*M*_ represents the wireless signal loss in the open area, and *f* is the frequency of the radio signal. *d* is the distance from the radio signal transmitting base station to the receiving end, the unit of this distance is km, *h*_*T*_ is the height of the transmitting antenna of the signal base station, *h*_*R*_ is the antenna height of the wireless signal receiving end, and the units of *h*_*R*_ and *h*_*T*_ are *m*. At the same time, *L*_free_ is the loss of free-space propagation of electromagnetic waves under ideal conditions, and *A*_*m*_ is the path loss in open poses. Moreover, *H*_*T*_ is the height gain factor of wireless signal transmission, *H*_*R*_ is the height gain factor of the antenna at the receiving end of the wireless signal, and the units of *H*_*T*_ and *H*_*R*_ are dB.

The article "Athlete Health Status Assessment Based on Edge Computing Model and Large-Scale Multimedia Health Data Analysis" was retracted in 2023. Reasons: signs of a paper mill; suspected computer-generated content; unreliable results or conclusions; concerns about the data.

However, it is typically difficult to create the optimum open pose state when dealing with real-world circumstances. In addition, the base stations that were chosen for this study are located in hilly and mountainous regions; as a result, the path propagation loss in the open pose cannot be directly employed, and the propagation loss in the open pose must be adjusted. In this study, the pose correction factor is added to the model of the path propagation loss for the open position pose. As a result, the path loss model for the complex pose is obtained as follows:

(16) $$\begin{array}{c} L_{M}=L_{\text{free}}+A_{m}\left(f,d\right)-H_{T}\left(h_{T},d\right)-H_{R}\left(h_{R},f\right)-k_{h}-k_{A}. \end{array}$$

Among them, *k*_*h*_ is the terrain correction parameter in the wave propagation loss, and *k*_*A*_ is the slope correction parameter in the propagation loss. A blockage in the wireless propagation path can be detected by adding these two correction parameters. The Okumura model's modified parameters can be used to determine this parameter. Using communication experiments, Okumura model's correction factors have been proven to be fairly accurate.

In addition, when the radio signal propagates in the sports field environment, the vegetation of the sports field will also attenuate the propagation of the wireless signal. In addition to the pose correction factor, the vegetation correction factor also needs to be added, and the loss model is obtained as

(17) $$\begin{array}{c} L_{M}=L_{\text{free}}+A_{m}\left(f,d\right)-H_{T}\left(h_{T},d\right)-H_{R}\left(h_{R},f\right)-k_{h}-k_{A}-k_{F}. \end{array}$$

Among them, *k*_*F*_ is the sports field correction factor. In order to establish a highly reliable near-Earth communication link, these attenuation effects must be considered. In a sports field, the relationship between signal propagation loss and distance and antenna height can be expressed by formula (18).

(18) $$\begin{array}{c} k_{F}=-20\;\log_{10}\left(h_{T}\right)-20\;\log\left(h_{R}\right)-20\;\log_{10}\left(\frac{3R_{0}}{2R}F_{s}F_{j}\right). \end{array}$$

In the formula, *R*_0_ is the radiation resistance of the dipole antenna in free space, and *R* is the total antenna resistance near the ground and leaves. Meanwhile, *F*_*s*_ is the factor affected by the curvature of the earth, *F*_*j*_ is the factor affected by the jungle, and *h*_*T*_, *h*_*R*_ are the height of the transmitting and receiving antennas, respectively. Finally, according to the Okumura model and actual empirical values, as well as the engineering application in the project, we obtain the empirical formula of the wireless signal propagation loss model in the irregular pose area under the influence of vegetation:

(19) $$\begin{array}{c} L_{M}=69.55+26.12\log_{10}\;f-13.82\log_{10}h_{T}\\ -R\left(h_{R}\right)+\left(44.9-6.55\;\log_{10}h_{T}\right)\log_{10}\;d. \end{array}$$

Among them, *R*(*h*_*R*_) is the correction parameter in hilly and mountainous areas, and the calculation formula of *R*(*h*_*R*_) in the experimental environment of this paper is as follows:

(20) $$\begin{array}{c} R\left(h_{R}\right)=\left(1.1\;\log_{10}\;f-0.7\right)h_{R}-\left(1.56\;\log_{10}\;f-0.8\right). \end{array}$$

After the propagation loss model under the irregular pose is obtained, the wireless signal power *P*_*R*_ received by the wireless signal receiver can be finally obtained:

(21) $$\begin{array}{c} P_{R}=P_{T}-L_{M}+G_{T}+G_{R}. \end{array}$$

Among them, *P*_*R*_ and *P*_*T*_ are the signal power received by the radio receiving end and the signal power transmitted by the radio transmitting end, and *G*_*T*_ and *G*_*R*_ are the antenna gains of the radio signal transmitting end and the receiving end, respectively.

The article "Athlete Health Status Assessment Based on Edge Computing Model and Large-Scale Multimedia Health Data Analysis" was retracted in 2023. Reasons: signs of a paper mill; suspected computer-generated content; unreliable results or conclusions; concerns about the data.

For a two-dimensional plane, the Euclidean distance formula is

(22) $$\begin{array}{c} D_{i}=\sqrt{{\left(X-X_{i}\right)}^{2}+{\left(Y-Y_{i}\right)}^{2}}. \end{array}$$

Among them, (*X*, *Y*) is the two-dimensional coordinate of the current node, and (*X*_*i*_, *Y*_*i*_) is the two-dimensional coordinate of the neighbor node.

The following is a detailed analysis of the forwarding situation of data packets in greedy forwarding. In a two-dimensional plane, the distribution of nodes is shown in Figure 1. In the Figure 1, *x* is the source node, *D* is the destination node, and the communication radius of the *x* node is shown by the dotted circle in Figure 1. As can be seen from Figure 1, there are multiple nodes within the communication range of node *x*, and they are all neighbor nodes of node *x*. However, node *y* is the closest to the destination node. Based on the idea of the greedy algorithm, the *x* node will use the *y* node as the next hop node. Based on this method, the data packet is finally sent from the source node to the destination node.

However, there are also problems with the two-dimensional greedy algorithm, as shown in Figure 2. In Figure 2, the distance between the source node *x* and the destination node is greater than the communication radius of the node, so one-hop forwarding cannot be performed directly. However, the distance between the neighbor node and the destination node is greater than the distance between itself and the destination node. Therefore, in this case, node *x* will not forward the packet to node *w* or node *y*.

The article "Athlete Health Status Assessment Based on Edge Computing Model and Large-Scale Multimedia Health Data Analysis" was retracted in 2023. Reasons: signs of a paper mill; suspected computer-generated content; unreliable results or conclusions; concerns about the data.

When the two-dimensional greedy forwarding algorithm encounters the routing hole problem, it cannot be solved by the greedy algorithm alone. At this time, the peripheral forwarding strategy is used to solve the problem. The core method of peripheral forwarding is the right-hand rule. The right-hand rule method is shown in Figure 3.

This paper conducts simulation experiments on greedy forwarding routing under two-dimensional conditions. The main purpose of the simulation test is to test the influence of the number of nodes on the route establishment in a certain area of the routing protocol based on two-dimensional greedy forwarding, including the number of hops of the route and the connectivity rate of the route.

First, the simulation conditions randomly generate several routing nodes in an area with a size of 100*∗*100, the communication radius of each node is 20, and a fixed source node and destination node are set. The simulation test is shown in Figure 4.

The simulation tests the effect of setting different number of nodes on the routing success rate when the area size is the same. The relationship between routing connectivity rate, hop count, and node density is shown in Figure 5 when the number of different nodes is obtained.

It can be seen from the experimental results that the routing success rate increases with the increase of node density. This is because the greater the node density is, the more nodes the route can choose to communicate with, and the higher the success rate is.

The simulation results of routing hops and node density are shown in Figure 6. From the relationship between the number of routing hops and node density, it can be seen that the number of routing hops decreases with the increase of node density. This is mainly because when the node density is low, the routing needs to perform multihop forwarding to complete the connection in order to connect. However, when the density increases, the node can choose the optimal node of the next hop to forward the data.

For the 3D greedy algorithm, the third dimension *z*-plane is also taken into account when doing the distance calculation. In the three-dimensional coordinate system, the Euclidean distance is calculated by the following formula:

(23) $$\begin{array}{c} D_{i}=\sqrt{{\left(X-X_{i}\right)}^{2}+{\left(Y-Y_{i}\right)}^{2}+{\left(Z-Z_{i}\right)}^{2}}. \end{array}$$

Among them, (*X*, *Y*, *Z*) is the 3D coordinate or pose coordinate of the current node whose neighbor list is being calculated. (*X*_*i*_, *Y*_*i*_, *Z*_*i*_) are the three-dimensional coordinates or pose coordinates of the nodes considered for neighbor selection. When *D*_*i*_ is smaller than the communication radius *R*, the target node is considered as a neighbor node.

The article "Athlete Health Status Assessment Based on Edge Computing Model and Large-Scale Multimedia Health Data Analysis" was retracted in 2023. Reasons: signs of a paper mill; suspected computer-generated content; unreliable results or conclusions; concerns about the data.

This paper simulates the relationship between the routing success rate and node density and the relationship between routing hops and node density when the two-dimensional greedy algorithm and the three-dimensional greedy algorithm are used.  Figure 7 is a three-dimensional greedy forwarding simulation environment.

In the simulation experiment, we set a 3D space of 100*∗*100*∗*100. The communication radius of each routing node is 20, the pose coordinates of the source node and the destination node are fixed, and several routing nodes are randomly generated in the three-dimensional space to test the actual effect of the two-dimensional greedy forwarding and the three-dimensional greedy forwarding in the three-dimensional space. Two-dimensional greedy forwarding only calculates the XY coordinates of the node in the three-dimensional space and only judges whether the node is within the communication range based on the XY coordinates. The 3D simulation is similar to the 2D simulation in that it tests the routing success rate and the relationship between routing hops and node density.

The relationship between the routing success rate and routing node density obtained by the simulation test is shown in Figure 8.

It can be seen from the simulation results that, with the increase of node density, the routing success rate of the 3D greedy algorithm also increases continuously. When the node density reaches 120/100^3^*m*^3^, the routing success rate can be stabilized at more than 90%. However, the improvement of the routing success rate of the two-dimensional greedy algorithm in the three-dimensional case is not significantly related to the improvement of the node density. It can be seen that the two-dimensional greedy algorithm cannot be directly used in the three-dimensional space.

The simulation results of the relationship between the number of routing hops and the node density of the 3D greedy algorithm are shown in Figure 9.

From the relationship between the number of routing hops and the density of nodes, it can be seen that, in the case of using three-dimensional greedy forwarding, the number of routing hops decreases with the increase of node density, and the number of routing hops of the three-dimensional greedy algorithm is significantly less than that of the two-dimensional greedy forwarding algorithm. It is not obvious that the number of routing hops of the two-dimensional greedy algorithm decreases with the increase of node density. It can be seen that the two-dimensional greedy forwarding algorithm is not suitable for the three-dimensional situation. The above results show that the three-dimensional greedy forwarding algorithm is more suitable for base station routing under realistic conditions.

The article "Athlete Health Status Assessment Based on Edge Computing Model and Large-Scale Multimedia Health Data Analysis" was retracted in 2023. Reasons: signs of a paper mill; suspected computer-generated content; unreliable results or conclusions; concerns about the data.

## 4. Athlete Health Status Assessment Based on Edge Computing Model and Large-Scale Multimedia Health Data Analysis

Figure 10 shows the framework of the athletes' health status assessment system based on the edge computing model in the large-scale multimedia health data analysis.

Figure 11 shows the real-time monitoring image of athletes' health status based on multimedia health data analysis and edge computing.

On the basis of the above analysis, the effect of the model proposed in this paper is verified, and the effect of the athlete health assessment system in this paper is counted, and the results are shown in Figure 12.

As can be seen from the aforementioned research, the athletes' health status assessment system that is proposed in this paper and is based on large-scale multimedia health data analysis and an edge computing model has a positive effect on athlete health assessment. This finding can be derived from the studies that were mentioned earlier.

## 5. Conclusion

Following an exhaustive review of the athlete's health state assessment report, which serves as the management component of the athlete's health management system, the athlete's health intervention program is a collection of intervention measures designed to effectively suppress and alleviate the athlete's health state. The goal of the top-level athlete's health management is to conduct an investigation into the factors that contribute to the subjects' current states of health. In addition, it plans the final athlete health improvement plan for the entire body by conducting an exhaustive and exhaustive evaluation of various inspection reports and the subject's behavior, lifestyle, eating habits, personality characteristics, mood, and living environment. This evaluation is done in order to arrive at the best possible plan for improving the athlete's health.

The purpose of this study is to investigate a system for assessing an athlete's health state that is based on the large-scale multimedia analysis of health data and the edge computing concept. The experimental analysis demonstrates that the athlete's health status assessment system suggested in this paper, which is based on large-scale multimedia health data analysis and an edge computing model, has a good effect on the assessment of athletes' health.

The article "Athlete Health Status Assessment Based on Edge Computing Model and Large-Scale Multimedia Health Data Analysis" was retracted in 2023. Reasons: signs of a paper mill; suspected computer-generated content; unreliable results or conclusions; concerns about the data.

## Figures and Tables

**Figure 1:** Schematic diagram of two-dimensional greedy forwarding mechanism.

**Figure 2:** Routing holes in greedy forwarding.

**Figure 3:** Right-hand rule.

**Figure 4:** Two-dimensional greedy forwarding simulation experiment.

**Figure 5:** Relationship between node density and routing success rate.

**Figure 6:** Relationship between node density and routing hops.

**Figure 7:** 3D greedy forwarding simulation experiment.

**Figure 8:** Relationship between node density and routing success rate under 3D simulation.

**Figure 9:** Relationship between routing hop count and node density.

**Figure 10:** Athlete health status assessment based on edge computing model and large-scale multimedia health data analysis.

**Figure 11:** Real-time monitoring images of athletes' health status. (a) Identification image of the athletes' health status. (b) Digitally processed image.

**Figure 12:** Effects of health assessment of athletes.

## Data Availability

The data used to support the findings of this study are included within the article.
